The article "Application of Whole-Body Hyperbaric Oxygen Therapy in the Treatment of Grade III Exposed Dog Bite Wounds" was published in 2022. Journal: Emerg Med Int.

# Application of Whole-Body Hyperbaric Oxygen Therapy in the Treatment of Grade III Exposed Dog Bite Wounds

**DOI:** 10.1155/2022/2570883

**Published:** 2022-09-21

**Authors:** Chao Tian, Qiang Yang, Shu-Zhen Bi, Xu-Rong Li, Jin-Hua Chen, Yao Guo

**Affiliations:** Department of Emergency, Changzhi People's Hospital, Changzhi 046000, China

## Abstract

**Objective:**

The aim of the study is to evaluate the therapeutic effect of hyperbaric oxygen in the treatment of grade III exposed dog bite wounds.

**Method:**

Fifty-two patients with grade III dog bite wounds who were seen in the emergency department of our hospital from 2017 to 2021 were selected for this research. The participants were randomly divided into an experimental group and a control group, with 26 patients in each group. The experimental group received hyperbaric oxygen therapy (HBOT), and the control group received routine treatment. The patients were followed up for three months after the treatment concluded. The wound healing rate, infection rate, and healing time were measured and compared.

**Results:**

The cure rate of the experimental group (96.2%) was higher than that of the control group (69.2%). The infection rate in the experimental group (3.8%) was lower than that of the control group (30.8%). The average cure time of the experimental group (9 ± 2.7) was lower than that of the control group (11 ± 3.4). The number of dressing changes in the experimental group (4 ± 3.0) was lower than that of the control group (7.5 ± 3.5), and there was a significant difference between the two groups (*P* < 0.05).

**Conclusion:**

According to the results, HBOT of grade III dog bite wounds can promote wound healing, improve the cure, and reduce the wound infection rate. It should have a primary role in the clinical treatment of these wounds.

## 1. Introduction

Dog bites are a common type of animal bite. Globally, nearly 100 million people are bitten by dogs every year [1]. Dog bites can cause skin damage, tissue tears, and infections [2]. Infection is the most common complication after a dog bite, primarily a mixed infection of aerobic and anaerobic bacteria [3]. Grade III exposed wounds are very common because the bite penetrates one or more skin layers, tissue damage occurs to at least the level of the dermis and blood vessels, and bleeding or subcutaneous tissue can be seen with the naked eye [4]. Therefore, it is very important to deal effectively with grade III exposed wounds caused by dog bites to avoid secondary bacterial infection and rabies [5].

Hyperbaric oxygen therapy (HBOT) involves exposing a patient to elevated gas pressure while they inhale pure oxygen. This method includes the use of a hyperbaric oxygen chamber, which can expose patients to 2 to 3 times the amount of normal gas pressure. This treatment method can be used for the primary or auxiliary treatment of infections such as gas gangrene, necrotizing fasciitis, diabetic foot infection, and refractory osteomyelitis, as well as neurosurgical and fungal infections [6]. The adjuvant treatment mechanism of HBOT may be related to the stimulation of angiogenesis, collagen synthesis, stem cells, and the local immune response. Domestic scholars report that hyperbaric oxygen assists in the treatment of various orthopedic and soft tissue infections of the limbs and satisfactory results have also been achieved for various postoperative complications [7].

The article "Application of Whole-Body Hyperbaric Oxygen Therapy in the Treatment of Grade III Exposed Dog Bite Wounds" was published in 2022. Journal: Emerg Med Int.

According to existing research, HBOT can improve blood circulation and reduce wound infection. It also has obvious anti-inflammatory and anti-infective effects and can quickly eliminate chronic inflammation in wound tissues [8, 9]. However, there are few studies on the use of hyperbaric oxygen in the treatment of dog bite wounds. Therefore, this study investigates HBOT as an intervention method to preliminarily explore its role in the treatment of dog bites and to provide methodological support for enriching dog bite intervention methods and improving the prognosis of patients.

## 2. Materials and Methods

### 2.1. General Information

The current study was conducted on patients treated from 2017 to 2021. A convenience sampling method was used, and the research participants included 52 patients with grade III exposed dog bite wounds who were treated in the emergency department of our hospital. Participants were randomly divided into an experimental group and a control group. This was done by creating 52 sealed envelopes (marked as the experimental group and control group, with 26 envelopes in each group). Each patient was handed an envelope randomly to divide them into one of the two groups. The experimental group received whole-body HBOT and the control group received routine treatment. Patient ages ranged from 2 to 83 years old (average: 42.35 ± 10.37 years). The participants included 25 males and 27 females. The inclusion criteria were as follows: (1) a grade III exposed dog bite wound was confirmed according to the rabies exposure grading standard [10] and (2) informed consent was provided by the patient or their family. The exclusion criteria were as follows: (1) patients with serious heart, liver, kidney, mental, and immune system diseases; (2) patients with systemic infection; (3) patients with tendon, nerve, blood vessel, and bone injuries and serious skin defects; (4) patients with a history of a food or drug allergy; (5) patients with other chronic diseases or malnutrition; and (6) the time from receiving the bite to arriving at the hospital was ≥24 h.

The article "Application of Whole-Body Hyperbaric Oxygen Therapy in the Treatment of Grade III Exposed Dog Bite Wounds" was published in 2022. Journal: Emerg Med Int.

### 2.2. Methods

The patients in the control group were treated according to dog bite treatment principles immediately after admission [10]. This treatment proceeded as follows: (1) the wound was washed thoroughly by first washing with 20% soapy water and flowing water for 15–20 min and then washing alternately with normal saline and 3% hydrogen peroxide until there was no soap or hydrogen peroxide residue remaining; (2) the skin was disinfected with 1% povidone-iodine solution from the wound to an area 5–8 cm away from the wound, and then the wound was disinfected with 0.05% povidone-iodine solution for 5 min before being scrubbed with normal saline; (3) surgical debridement was then carried out by exploring the wound depth and degree of soft tissue damage, removing inactive tissue, expanding the wound if necessary, completely stopping any bleeding, and locally infiltrating the wound with an antirabies immune serum; (4) immunization was carried out by injecting the rabies vaccine (and subsequent vaccine series according to the regulations) and tetanus antiviral toxin or tetanus immunoglobulin; and (5) antibiotics were used in cases that had confirmed infections. The head, face, and immunocompromised parts were injected with rabies immunoglobulin around the wound. The antibody infiltrated human tissues to neutralize the virus. The larger wound was infiltrated, and human rabies immunoglobulin was injected around the wound. It was loosely sutured 2 h after the specification, and drainage strips were placed if necessary.

The experimental group was treated with early and thorough debridement of the wound, negative pressure drainage, and if necessary, routine injection with a tetanus antitoxin, administration of a rabies vaccine, and early hyperbaric oxygen intervention. A Yc32110/0.3-20ivw fully automatic medical hyperbaric oxygen chamber (Yantai Binglun hyperbaric oxygen chamber Co., Ltd.) was used. Hyperbaric oxygen treatment was provided using a single hyperbaric oxygen chamber and pure oxygen at a pressure of 253 kpa (2.5 times atmospheric pressure). Treatment was delivered twice daily during the first week and once a day after one week for a total of two weeks, and broad-spectrum antibiotics were applied to treat the infection.

### 2.3. Observation Indicators

The cure rates, wound infection rates, wound healing times, and primary and dressing change times of the two groups were observed.

The main infection criteria included (at least one of) the following: fever (body temperature >38°C), formation of a local abscess, or lymphangitis. The secondary criteria (all four criteria at the same time) included the following: the redness range of the tissue around the wound edge exceeding 2 cm, tenderness around the wound, local swelling around the wound, purulent secretion, and white blood cells >12 × 10^9^/L [11].

The article "Application of Whole-Body Hyperbaric Oxygen Therapy in the Treatment of Grade III Exposed Dog Bite Wounds" was published in 2022. Journal: Emerg Med Int.

### 2.4. Statistical Treatment

Statistical analysis was carried out using SPSS statistical software 22.0. The measurement data were expressed by the mean ± standard deviation using a *t* test, and the counting data were expressed by *n* (%) using a chi-square test. The difference was considered statistically significant at *P* < 0.05.

## 3. Results

### 3.1. Comparison of the Basic Data of the Two Groups

There were 12 males and 14 females in the control group, with an average age of 33.42 years. There were 14 males and 12 females in the experimental group, with an average age of 38.71 years. There were 49 wounds in the control group, with an average wound diameter of 3.35 ± 2.15 cm and an average wound depth of 1.5 ± 0.3 cm. There were 53 wounds in the experimental group, with an average wound diameter of 3.42 ± 2.05 cm and an average wound depth of 1.4 ± 0.2 cm. There was no significant difference between the two groups (*P* > 0.05) See Table 1.

### 3.2. Comparison of Healing between the Two Groups

The wound healing rate was 96.2% in the experimental group and 69.2% in the control group. The difference between the two groups was statistically significant (*P* < 0.05). See Table 2.

### 3.3. Comparison of the Wound Infection Rate, Wound Healing Time, and Healing Degree between the Two Groups

The infection rate in the experimental group was 3.8%, which was lower than the 30.8% rate in the control group. The difference between the two groups was statistically significant (*P* < 0.05). The average cure time of the experimental group was 9 ± 2.7 days, which was lower than that of the control group (11 ± 3.4 days). The difference between the two groups was statistically significant (*P* < 0.05). The number of dressing changes in the experimental group was 4 ± 3.0, which was lower than the number of changes (7.5 ± 3.5) in the control group. There was a significant difference between the two groups (*P* < 0.01). See Table 3.

## 4. Discussion

A grade III exposed dog bite wound is a special type of surgical wound. Anaerobic bacteria and aerobic bacteria exist at the same time, and an avulsion injury is formed due to the dog's teeth penetrating the skin. In addition to tissue suppuration and infection, serious complications such as arthritis, local erysipelas, limb lymphangitis, and sepsis can occur [12]. The technical guide for rabies prevention and control (2016 Edition) [11] points out that there are two main objectives for dog bite wound treatment: one is to prevent the occurrence of rabies and the other is to prevent secondary bacterial infection of the wound and promote wound healing. Timely and correct wound cleaning and disinfection, vaccination with a standardized rabies vaccine, and injection of immunoglobulin are the main measures to be taken to prevent rabies and wound infection. Wounds infected with both bacteria and viruses require long-term healing [13]. Therefore, effective promotion of wound healing is vital for supporting a good prognosis See Figure 1.

The article "Application of Whole-Body Hyperbaric Oxygen Therapy in the Treatment of Grade III Exposed Dog Bite Wounds" was published in 2022. Journal: Emerg Med Int.

Hyperbaric oxygen treatment can significantly promote wound healing. Studies have shown that this treatment method can promote wound recovery, inhibit the inflammatory response, and promote functional recovery in the adjuvant treatment of brain trauma, limb trauma, spinal cord injury, and visceral injury [14–16]. In terms of animal bites, HBOT has been applied to the adjuvant treatment of toxic animal bites, including snakes and spiders, with good results [17–19]. In the current study, 52 patients with grade III exposed dog bite wounds were selected and randomly divided into an HBOT treatment group and a standard method treatment control group. The results showed that compared with the control group, patients treated with HBOT had better results in terms of cure rate, wound infection rate, and cure time. Anaerobic bacteria exist in dog bite wounds, and more than 50% of the infections in these wounds are caused by these anaerobic bacteria [18, 19]. Oxygen therapy not only creates an oxygen-enriched environment around the wound that inhibits the anaerobic bacteria but also improves the ability of tissue regeneration and accelerates capillary regeneration [20]. Therefore, hyperbaric oxygen was used in this study. The results showed that HBOT could prevent wound infection and shorten the time of wound bed preparation. Bin et al. [21] also demonstrated that the combined oxygen treatment of pressure-ulcer-infected wounds can reduce the number of bacteria and reduce the probability of wound infection.

Good recovery, especially primary healing, reflects the overall promotion of patients' health. This not only is conducive to functional recovery but also has a positive impact on patients' psychological and social relations. A reduced healing time helps patients return to society faster and greatly reduces the risks associated with the wound-healing process. This effect is reflected in other findings in this study. The results showed that the wound infection rate and dressing change times in the experimental group were significantly lower than those in the control group. A lower dressing change time effectively avoids friction to the wound due to the reduced number of dressing changes and reduces the damage to the wound tissue; therefore, the prognosis is better and there is less scarring. This is not only related to the impact of HBOT itself; [22] shortened healing time also plays an important role in this regard.

The article "Application of Whole-Body Hyperbaric Oxygen Therapy in the Treatment of Grade III Exposed Dog Bite Wounds" was published in 2022. Journal: Emerg Med Int.

Although most studies support the notion that HBOT can accelerate the wound healing process, it is difficult to compare clinical trials in terms of hyperbaric oxygen use, primarily due to the heterogeneity of experimental designs, the injury types involved, and the outcome evaluations. A limitation of this study was the small number of samples, which may have resulted in a selection bias. However, since only a few similar studies are currently available, this study still presents results indicative of significance and can be used as a precursor for additional in-depth research.

## 5. Conclusion

Hyperbaric oxygen can promote the healing of dog bite wounds, greatly reduce wound infection, and shorten wound healing time. Therefore, its internal mechanism and specific effects are worthy of further research.

## Figures and Tables

**Figure 1:** Recovery of patients with different treatment methods. a–d represent patients in the hyperbaric oxygen intervention group. The patients showed open injuries (a, c) and healed well after intervention (b, d); e–h represent patients in the general treatment control group. The injured parts (e, g) of the patients were not completely healed after treatment (f, h).

**Table 1:** Comparison of basic data between the two groups.

Characteristics	Control group	Experimental group	*χ* ^2^ * /t*	*P*
*Gender*				
Male	12	14	0.317	0.574
Female	14	12		
Average age (years)	33.42 ± 3.37	38.71 ± 2.45	0.974	0.338
Number of wounds	49	53	0.312	0.826
Wound diameter	3.35 ± 2.15	3.42 ± 2.05	0.118	0.907
Wound depth	1.5 ± 0.3	1.4 ± 0.2	0.850	0.400

**Table 2:** Comparison of primary healing rate between the two groups.

Group	Number of wounds with primary healing	Number of wounds	Composition ratio (%)	*P*
Control group	26	49	53.1	0.024
Experimental group	39	53	73.6	

**Table 3:** Comparison of wound infection rate, healing time, and dressing change between the two groups of patients.

Group	Wound infection rate (%)	Healing time (d)	Number of dressing changes	Healing rate (%)
Control group	30.8	11 ± 3.4	7.5 ± 3.5	69.2%
Experimental group	3.8^*∗*^	9 ± 2.7^*∗*^	4 ± 3.0^*∗∗*^	96.2^*∗*^

^*∗*^ *P* < 0.05 compared with the control group; ^*∗∗*^*P* < 0.01 compared with the control group. The patient wound infection rate was compared using the adjusted *χ*^2^ test, and the healing time and the number of dressing changes were tested using the rank sum test of independent samples.

The article "Application of Whole-Body Hyperbaric Oxygen Therapy in the Treatment of Grade III Exposed Dog Bite Wounds" was published in 2022. Journal: Emerg Med Int.

## Data Availability

The datasets used or analyzed during the current study are available from the corresponding author upon reasonable request.
